The article "Efficacy of TACE+Radiofrequency Ablation+Sorafenib in the Treatment of Patients with Recurrent Liver Cancer and Construction of Prediction Model" was retracted in 2023. Reasons: signs of a paper mill; compromised peer review; unreliable results or conclusions.

# Efficacy of TACE+Radiofrequency Ablation+Sorafenib in the Treatment of Patients with Recurrent Liver Cancer and Construction of Prediction Model

**DOI:** 10.1155/2022/6879035

**Published:** 2022-09-07

**Authors:** Aimin Sun, Shumei Chen, Minggang Lin, Dapeng Zhou, Hongyan Zhang, Cheng Sun, Pan Wang

**Affiliations:** ^1^Department of Oncology, Qingdao Chengyang District People's Hospital, Qingdao, Shandong 226001, China; ^2^Department of Outpatient, Qingdao Chengyang District People's Hospital, Qingdao, Shandong 226001, China; ^3^Department of Interventional Medicine, Qingdao University, Qingdao, Shandong 226001, China; ^4^Department of 3D Medical Printing Center, Qingdao Chengyang District People's Hospital, Qingdao Shandong 226001, China

## Abstract

**Objective:**

This study is aimed at exploring the efficacy of transarterial chemotherapy embolization (TACE)+radiofrequency ablation+sorafenib in the treatment of patients with recurrent liver cancer and at constructing its prediction model.

**Methods:**

A total of 60 patients with recurrent liver cancer treated in our hospital from March 2020 to March 2022 were enrolled and divided into two groups according to treatment methods, with 30 patients in each group. Group A adopted TACE+radiofrequency ablation+sorafenib therapy while group B adopted TACE+radiofrequency ablation therapy. Clinical efficacy, complications, and adverse reactions of the two groups were observed. A total of 30 patients with nonrecurrent liver cancer in the same period were enrolled. 60 patients with recurrent liver cancer and 30 patients with nonrecurrent liver cancer were taken as the recurrence group and the nonrecurrence group, respectively. The baseline data and clinical data of the patients were queried by the Hospital Information System. The data included age, gender, Child-Pugh grade, HBV/HCV infection, portal vein tumor thrombus, degree of differentiation, vascular invasion, serum alpha fetal protein (AFP) level, number of tumors, maximum diameter of tumors, and number of nodules. The logistic regression analysis was used to analyze the independent risk factors for liver cancer recurrence. The Hosmer-Lemeshow test was used to analyze the degree of fitting between the prediction model and the standard curve. The ROC curve was used to analyze the predictive value of the model for liver cancer recurrence.

**Results:**

The objective effective rate and disease control rate in group A (33.33% and 70.00%) were higher than those in group B (10.00% and 43.33%), and the differences were statistically significant (both *P* < 0.05). There were no significant differences in the incidence of complications such as embolism syndrome, hand and foot skin reaction, gastrointestinal reaction, hypertension, diaphragmatic injury and bleeding, and biliary leakage and fever between the two groups (all *P* > 0.05). The proportions of patients in the recurrence group with portal vein tumor thrombus (PVTT), medium and high degree of differentiation, combined with vascular invasion, serum AFP level ≥ 400 ng/dL, multiple tumors, maximum tumor diameter ≥ 5 cm, combined with cirrhosis, and polynodules were all higher than those in the nonrecurrence group; the differences were statistically significant (all *P* < 0.05). Complication of PVTT, the degree of medium and high differentiation, and the maximum tumor diameter ≥ 5 cm were independent risk factors for recurrence of liver cancer (all *P* < 0.05). The prediction model of liver cancer recurrence was obtained by multiple regression analysis, *P* = 1/[1 + *e*^−(−5.441 + 6.154∗PVTT + 3.475∗differentiateddegree + 3.001∗maximumdiameteroftumor)^]. The Hosmer-Lemeshow test showed that *χ*^2^ = 1.558 (*P* = 0.992). According to the ROC curve analysis, the AUC, SE, and 95% CI value of the prediction model for liver cancer recurrence were 0.977, 0.012, and 0.953-1.000, respectively.

The article "Efficacy of TACE+Radiofrequency Ablation+Sorafenib in the Treatment of Patients with Recurrent Liver Cancer and Construction of Prediction Model" was retracted in 2023. Reasons: signs of a paper mill; compromised peer review; unreliable results or conclusions.

**Conclusion:**

TACE+radiofrequency ablation+sorafenib is effective in the treatment of recurrent liver cancer, and the prediction model established based on the risk factor has high predictive value for patients with recurrent liver cancer.

## 1. Introduction

Primary liver cancer (PLC) is a common malignant tumor disease in clinical practice. Its mortality and morbidity of liver cancer rank the second and third, respectively, among all malignant tumor diseases, and its morbidity is relatively high in Asia [1, 2]. PLC includes intrahepatic bile duct carcinoma, hepatocellular carcinoma (HCC), and bile duct carcinoma. At present, radical therapies for PLC mainly include complete tumor resection and liver transplantation. Due to the serious shortage of liver transplantation donors, hepatectomy is still the first-line treatment for most PLC patients with good liver function reserve. However, the recurrence rate of PLC is still as high as 50%-70% within 5 years after surgery. Recurrence and metastasis after surgical resection can seriously affect the long-term survival and quality of life of PLC patients. Although a variety of adjuvant therapies are also used clinically to reduce postoperative recurrence, the effect is not satisfactory and needs to be further explored [3, 4]. At present, the main clinical treatment methods for patients with recurrent liver cancer include resectomy, transarterial chemotherapy embolization (TACE), targeted therapy, local ablation, radiofrequency ablation, and salvage liver transplantation. Hepatectomy is the gold standard for the treatment of recurrent liver cancer. However, hepatectomy is faced with problems such as acute liver failure and insufficient liver function reserve due to the small size of the liver after resection, and only 6%~31% of patients can be resected again. Radiofrequency ablation and repeated resection have similar survival rates. TACE and radiofrequency ablation are both effective methods for the treatment of recurrent liver cancer. Sorafenib is an oral multikinase inhibitor that prolongates survival of patients with advanced liver cancer. Sorafenib is a targeted therapy. The purpose of this study was to explore the effect of TACE+radiofrequency ablation+sorafenib in the treatment of patients with recurrent liver cancer and to provide reference for the prevention and treatment of recurrent liver cancer by constructing a prediction model for liver cancer recurrence. The report is as follows.

The article "Efficacy of TACE+Radiofrequency Ablation+Sorafenib in the Treatment of Patients with Recurrent Liver Cancer and Construction of Prediction Model" was retracted in 2023. Reasons: signs of a paper mill; compromised peer review; unreliable results or conclusions.

## 2. Data and Methods

### 2.1. General Data

A total of 60 patients with recurrent liver cancer treated in our hospital from March 2020 to March 2022 were enrolled and divided into group A and group B according to treatment methods, with 30 patients in each group. In group A, there were 19 males and 11 females. The age ranged from 39 to 64 years, with the average age of 54.30 ± 6.28 years. Complications included hypertension in 8 cases, diabetes in 3 cases, and others in 19 cases. In group B, there were 17 males and 13 females. The age range was 39-77 years, with an average of 55.43 ± 10.79 years. Complications included hypertension in 12 cases, diabetes in 5 cases, and others in 13 cases. During the same period, a total of 30 patients with nonrecurrent liver cancer were enrolled as the nonrecurrence group. There were 18 males and 12 females. The age range was 38-72 years, with an average of 55.36 ± 7.52 years. Complications included hypertension in 10 cases, diabetes in 4 cases, and others in 16 cases. The general data of the three groups were comparable (all *P* > 0.05). This study was approved by the Hospital Ethics Committee.

### 2.2. Inclusion Criteria

The inclusion criteria of this study are as follows: (1) age > 18, (2) all patients were diagnosed with recurrent liver cancer by clinicopathological diagnosis, (3) the maximum diameter of the tumor was 1-7 cm, (4) the life expectancy > 3 months, and (5) all patients participated in this study voluntarily.

### 2.3. Exclusion Criteria

The exclusion criteria of this study are as follows: (1) patients with other malignant tumor diseases, (2) patients with Child-Pugh grade C for liver function, (3) patients with severe organ dysfunction such as heart, lung, and kidney, (4) patients who cannot tolerate TACE and radiofrequency ablation or were allergic to sorafenib, and (5) patients with severe coagulation dysfunction that were uncorrectable.

The article "Efficacy of TACE+Radiofrequency Ablation+Sorafenib in the Treatment of Patients with Recurrent Liver Cancer and Construction of Prediction Model" was retracted in 2023. Reasons: signs of a paper mill; compromised peer review; unreliable results or conclusions.

### 2.4. Methods

Group A was treated with TACE+radiofrequency ablation+sorafenib, and group B was treated with TACE+radiofrequency ablation.

#### 2.4.1. TACE

The femoral artery was punctured with Seldinger technique routinely, and the 5F catheter was placed. The catheter was placed at the opening of the celiac trunk artery for angiography to determine the tumor target vessel. Superselective intubation was performed into the tumor supplying artery. The tumor target vessel was embolized with fluorouracil 1000 mg, cisplatin 50 mg, pirarubicin 50 nmg+super liquefied lipiodol 5~10 mL. After the operation, hepatoprotective hydration treatment was performed.

#### 2.4.2. Radiofrequency Ablation

After the TACE treatment for 2-4 weeks, radiofrequency ablation was performed. First, CT scanning was performed to determine the puncture point, and then, lidocaine was used for local anesthesia. Percutaneous puncture of intrahepatic lesions was performed under the guidance of the CT, and tumor ablation was performed according to the protocol. After that, CT scanning was performed to see whether the scope covered the target tumor. If it was not completely covered, radiofrequency ablation could be performed immediately. During radiofrequency ablation, all lesions should be ablated in one ablation process, including single nodule and polynodule patients.

#### 2.4.3. Sorafenib Treatment

Seven days after intervention, sorafenib was given orally, 400 mg/time, twice a day for 4 weeks.

### 2.5. Observation Indicators

(1) The clinical efficacy of group A and group B was evaluated according to the efficacy evaluation criteria. (2) There is a comparison of complication rate between group A and group B. (3) A total of 30 patients with nonrecurrent liver cancer in the same period were selected, and 60 patients with recurrent liver cancer and 30 patients without recurrent liver cancer were divided into the recurrence group and the nonrecurrence group. The baseline data and clinical data of patients were queried by hospital information system. Age, gender, Child-Pugh grade, HBV/HCV infection, portal vein tumor thrombus, differentiation degree, vascular invasion, serum AFP level, tumor number, tumor maximum diameter, number of nodules, and other data were included. Baseline data and clinical data were compared between the recurrence group and the non-recurrence group. (4) Logistic multivariate regression analysis was used to analyze the independent risk factors of HCC recurrence. The baseline and clinical data of the recurrence group and the nonrecurrence group were statistically different. (5) Logistic regression was used to analyze the risk factors of HCC recurrence and establish a regression model. (6) The receiver operating characteristic (ROC) curve was used to calculate the discrimination of the prediction model.

The article "Efficacy of TACE+Radiofrequency Ablation+Sorafenib in the Treatment of Patients with Recurrent Liver Cancer and Construction of Prediction Model" was retracted in 2023. Reasons: signs of a paper mill; compromised peer review; unreliable results or conclusions.

### 2.6. Efficacy Evaluation Criteria

The treatment effects of the two groups were assessed according to the Response Evaluation Criteria in Solid Tumors (RECIST) [5] proposed by the American Cancer Institute. The treatment effects were divided into complete remission (CR), partial remission (PR), stable disease (SD), progressive disease (PD), objective response rate (ORR) = CR + PR, and disease control rate (DCR) = CR + PR + SD.

### 2.7. Statistical Method

All the data in this study were entered into Excel form without communication between two persons and analyzed and processed with statistical software SPSS 24.0. The measurement data were expressed in mean ± SD (±*s*). When the measurement data conform to the normal distribution and the variance was homogeneous, a *t*-test was adopted. The counting data were described by *N* and %. The disordered classification data were compared by the *χ*^2^ test or Fisher's exact probability method. The logistic regression analysis was used to analyze the risk factors of liver cancer recurrence. The Hosmer-Lemeshow test was used to analyze the fitting degree between the prediction model and the standard curve. The ROC curve was used to analyze the predictive value of the model for recurrence of liver cancer. All tests were two-sided, and the difference was statistically significant when *P* < 0.05.

## 3. Results

### 3.1. Comparison of Clinical Efficacy between the Two Groups

The ORR and DCR in group A (33.33% and 70.00%) were higher than those in group B (10.00% and 43.33%). The differences were statistically significant (both *P* < 0.05, Table 1).

### 3.2. Comparison of Complications and Adverse Reactions between the Two Groups

There were no significant differences in the incidence of complications such as embolism syndrome, hand and foot skin reaction, gastrointestinal reaction, hypertension, diaphragmatic injury and bleeding, and biliary leakage and fever between the two groups (all *P* > 0.05) as shown in Table 2.

### 3.3. Univariate Analysis of Recurrence in Two Groups

The proportion of patients in the recurrence group with PVTT, medium and high degree of differentiation, combined with vascular invasion, serum AFP level ≥ 400 ng/dL, multiple tumors, maximum diameter ≥ 5 cm, combined with cirrhosis, and polynodules was higher than that in the nonrecurrence group; the differences were statistically significant (all *P* < 0.05), as shown in Table 3.

The article "Efficacy of TACE+Radiofrequency Ablation+Sorafenib in the Treatment of Patients with Recurrent Liver Cancer and Construction of Prediction Model" was retracted in 2023. Reasons: signs of a paper mill; compromised peer review; unreliable results or conclusions.

### 3.4. Logistic Multivariate Analysis of Recurrence in Two Groups

Complication of PVTT, the degree of medium and high differentiation and the maximum tumor diameter ≥ 5 cm were independent risk factors for recurrence of liver cancer (all *P* < 0.05), as shown in Table 4.

### 3.5. Establishment of Prediction Model and Analysis of Model Calibration Degree

The predictive model of liver cancer recurrence was obtained by multiple regression analysis, *P* = 1/[1 + *e*^−(−5.441 + 6.154∗PVTT + 3.475∗Degreeofdifferentiation + 3.001∗Maximumdiameteroftumor)^]. The Hosmer-Lemeshow test showed that *χ*^2^ = 1.558 and *P* = 0.992 (Figure 1).

### 3.6. Prediction Efficiency Analysis of Prediction Model

According to ROC curve analysis, the AUC value, SE value, and 95% CI of the prediction model for HCC recurrence were 0.977, 0.012, and 0.953-1.000, respectively (Figure 2).

## 4. Discussions

Most recurrent liver cancer cannot tolerate secondary surgery because of specific tumor location, multiple recurrent foci, and complicated with severe cirrhosis. TACE is the preferred treatment for nonsurgical treatment of recurrent liver cancer [6–8]. TACE technology combines embolization and chemotherapy. Chemotherapy drugs can be injected through the hepatic artery to increase drug concentration in tumor tissue and reduce side effects of systemic chemotherapy. The use of iodized oil to suspend chemotherapy drugs can concentrate the drug in tumor tissue. Transcatheter therapy for liver cancer allows direct delivery of embolic agents to the liver tumor, preserving normal liver tissue, and promoting the absorption of drugs into cancer cells [9–11]. Radiofrequency ablation is considered to be a radical treatment strategy for PLC comparable to liver resection and liver transplantation, with the advantages of repeatable operation, less trauma and fewer complications. In addition to PLC, radiofrequency ablation can be applied to single or relatively limited intrahepatic recurrence to improve the long-term outcomes of patients [12, 13]. *Guidelines for the Diagnosis and Treatment of Primary Liver Cancer (2022)* [14] indicates that radiofrequency ablation is suitable for liver cancer patients with single tumor with diameter ≤ 5 cm, multiple tumors with maximum tumor with diameter ≤ 3 cm, tumor nodules with diameter ≤ 3 cm, no vascular invasion, and distant metastasis. For patients with single or multiple tumors that cannot be treated surgically, TACE combined with radiofrequency ablation can be used. Sorafenib is a molecular targeted drug, a multikinase inhibitor, which can effectively prolong the survival time of liver cancer patients. In addition, according to relevant studies, sorafenib can expand the range of radiofrequency ablation and improve the therapeutic effect of liver cancer treatment [15]. Treating liver cancer with TACE alone also has some limitations. TACE treatment of liver cancer can cause anoxic environment, induced VEGF expression, and neovascularization, while TACE combined with sorafenib to treat liver cancer can effectively inhibit regenerating blood vessels, reduce tumor recurrence and metastasis, and improve the therapeutic effect. In this study, the ORR and DCR of group A (33.33% and 70.00%) after treatment were higher than that of group B (10.00% and 43.33%) (both *P* < 0.05). Group A was given TACE+radiofrequency ablation+sorafenib, and group B was given TACE+radiofrequency ablation. These results indicated that the combination of TACE+radiofrequency ablation+sorafenib was more effective in the treatment of recurrent liver cancer, which may be related to the synergistic therapeutic effect of sorafenib with TACE and radiofrequency ablation. There were no significant differences in the incidence of complications such as embolism syndrome, hand and foot skin reaction, gastrointestinal reaction, hypertension, diaphragmatic injury and bleeding, and biliary leakage and fever between the two groups (all *P* > 0.05). Although sorafenib was added in group A, there was no increase in the incidence of serious adverse reactions and complications indicating that sorafenib are safe for treatment.

The article "Efficacy of TACE+Radiofrequency Ablation+Sorafenib in the Treatment of Patients with Recurrent Liver Cancer and Construction of Prediction Model" was retracted in 2023. Reasons: signs of a paper mill; compromised peer review; unreliable results or conclusions.

Comparison of baseline and clinical data between the two groups showed that the proportion of patients in the recurrence group with PVTT, medium and high degree of differentiation, combined with vascular invasion, serum AFP level ≥ 400 ng/dL, multiple tumors, maximum diameter ≥ 5 cm, combined with cirrhosis, and polynodules was significantly higher than that in the nonrecurrence group (all *P* < 0.05). The results showed that the complication of PVTT, medium and high degree of differentiation, vascular invasion, serum AFP level ≥ 400 ng/dL, multiple tumors, maximum tumor diameter ≥ 5 cm, cirrhosis, and polynodules were related to the recurrence of liver cancer. The recurrence of liver cancer is generally caused by multicentric canceration, and the high recurrence rate after surgery also seriously affects the therapeutic effect. Early recurrence was mainly related to tumor size, vascular invasiveness, and higher AFP level in muscle serum of the primary tumor, while late recurrence was mainly related to etiology and cirrhosis background. Vascular invasion can lead to worse tumor stage and tumor progression in patients, and PVTT is a common complication in patients with liver cancer, indicating poor prognosis [16]. Tumor grade can significantly affect the independent influencing factors of long-term survival, and the histological grade of tumor can represent the biological aggressiveness of liver cancer. Multiple previous studies have shown that tumor grade is a negative prognostic indicator [17, 18], which is consistent with the results of our study. Serum AFP indicators play an important role in early detection, and serum AFP level can be used as an independent predictor of overall survival before salvage treatment, and a higher AFP level indicates a higher degree of malignancy of liver cancer [19]. The number and maximum diameter of tumors are related to the early recurrence of liver cancer. Large liver cancer with a diameter of >5 cm is highly invasive and has a high risk of recurrence, which may be related to large tumor size, compression or invasion of large blood vessels. Previous studies have also shown that cirrhosis and polynodules are risk factors for liver cancer recurrence [20–22]. The logistic multivariate analysis showed that PVTT, medium and high differentiation degree, and maximum tumor diameter ≥ 5 cm were independent risk factors for liver cancer recurrence (all *P* < 0.05). PVTT, serum AFP level ≥ 400 ng/dL, multiple tumors, cirrhosis, and polynodular were not the independent risk factors for liver cancer recurrence. This result may be related to the small number of cases in this study.

The article "Efficacy of TACE+Radiofrequency Ablation+Sorafenib in the Treatment of Patients with Recurrent Liver Cancer and Construction of Prediction Model" was retracted in 2023. Reasons: signs of a paper mill; compromised peer review; unreliable results or conclusions.

The identification of patients with recurrent liver cancer by predictive model is conducive to the timely intervention by clinicians and the development of individualized control programs for high risk factors, which is conducive to further reducing the recurrence rate of liver cancer and improving the prognosis of liver cancer patients. In this study, a prediction model was established based on various risk factors. The Hosmer-Lemeshow test and ROC curve analysis showed that the model had high predictive value for liver cancer recurrence and could be used in the early prediction of liver cancer recurrence.

In conclusion, TACE+radiofrequency ablation+sorafenib has a good clinical effect in the treatment of recurrent liver cancer, and the prediction model established based on risk factors has a high predictive value for the recurrence of liver cancer.

## Figures and Tables

**Figure 1:** Analysis of model calibration degree.

**Figure 2:** ROC curve analysis of prediction model for predicting liver cancer recurrence.

**Table 1:** Comparison of clinical efficacy between the two groups [*n* (%)].

Group	CR	PR	SD	PD	ORR	DCR
Group A (*n* = 30)	1 (3.33)	9 (30.00)	11 (36.67)	9 (30.00)	10 (33.33)	21 (70.00)
Group B (*n* = 30)	0 (0.00)	3 (10.00)	10 (33.33)	17 (56.67)	3 (10.00)	13 (43.33)
*χ* ^2^-value					4.812	4.344
*P* value					0.028	0.037

CR: complete remission; PR: partial remission; SD: stable disease; PD progressive disease; ORR: objective response rate; DCR: (disease control rate).

The article "Efficacy of TACE+Radiofrequency Ablation+Sorafenib in the Treatment of Patients with Recurrent Liver Cancer and Construction of Prediction Model" was retracted in 2023. Reasons: signs of a paper mill; compromised peer review; unreliable results or conclusions.

**Table 2:** Comparison of complications and adverse reactions between the two groups [*n* (%)].

Group	Embolism syndrome	Hand-foot skin reaction	Gastrointestinal reaction	Hypertension	Diaphragm injury and bleeding	Biliary leakage and fever
Group A (*n* = 30)	28 (93.33)	23 (76.67)	27 (90.00)	9 (30.00)	12 (40.00)	10 (33.33)
Group B (*n* = 30)	27 (90.00)	21 (70.00)	23 (76.67)	12 (40.00)	10 (33.33)	7 (23.33)
*χ* ^2^-value		0.341	1.920	0.659	0.287	0.739
*P* value		0.559	0.166	0.417	0.592	0.390
Fisher's exact probability value	1.000					

**Table 3:** Univariate analysis of recurrence in two groups [$\bar{x}\pm s$, *n* (%)].

Item	Recurrence group (*n* = 60)	Nonrecurrence group (*n* = 30)	*χ* ^2^ value	*P* value
Age (years)				
<60 years	37 (61.67)	18 (60.00)	0.023	0.878
≥60 years	23 (38.33)	12 (40.00)		
Gender				
Male	36 (60.00)	20 (66.67)	0.378	0.539
Female	24 (40.00)	10 (33.33)		
Child-Pugh grade				
Grade A	44 (73.33)	17 (56.67)	2.544	0.111
Grade B	16 (26.67)	13 (43.33)		
HBV/HCV infection				
No	39 (65.00)	14 (46.67)	2.777	0.096
Yes	21 (35.00)	16 (53.33)		
PVTT				
Yes	52 (86.67)	2 (6.67)	53.33	<0.001
No	8 (13.33)	28 (93.33)		
Degree of differentiation				
High differentiation	17 (28.33)	4 (13.33)	8.921	0.012
Medium differentiation	28 (46.67)	9 (30.00)		
Low differentiation	15 (25.55)	17 (56.67)		
Vascular invasion				
Yes	28 (46.67)	3 (10.00)	11.908	0.001
No	32 (53.33)	27 (90.00)		
Serum AFP level (ng/dl)				
<400	22 (36.67)	18 (60.00)	4.410	0.036
≥400	38 (63.33)	12 (40.00)		
Number of tumors				
Single	27 (54.00)	23 (76.67)	8.122	0.004
Multiple	33 (82.50)	7 (23.33)		
Maximum diameter of tumor (cm)				
<5	29 (48.33)	22 (73.33)	5.090	0.024
≥5	31 (51.67)	8 (26.67)		
Cirrhosis				
Yes	24 (40.00)	19 (63.33)	4.364	0.037
No	36 (60.00)	11 (36.67)		
Number of nodules				
Single nodule	25 (41.67)	20 (66.67)	5.000	0.025
Polynodule	35 (58.33)	10 (33.33)		

**Table 4:** Logistic multivariate analysis of recurrence in two groups.

Item	*β*	*SE*	Wald *χ*^2^	OR	95% CI	*P* value
PVTT	6.154	1.710	12.947	470.733	16.477~13448.349	< 0.001
Degree of differentiation	3.475	1.475	5.548	32.295	1.792~581.983	0.019
Vascular invasion	1.636	1.212	1.822	5.134	0.477~55.220	0.177
Serum AFP level (ng/dL)	1.705	1.151	2.196	5.502	0.577~52.479	0.138
Number of tumors	0.940	1.196	0.617	2.560	0.245~26.695	0.432
Maximum diameter of tumor	3.001	1.520	3.898	20.109	1.022~395.55	0.048
Cirrhosis	-2.997	1.587	3.566	0.050	0.002~1.120	0.059
Number of nodules	0.928	1.138	0.665	2.531	0.272~23.557	0.415
Constant	-5.441	1.857	8.581	0.004		0.003

PVTT: yes = 1 and no = 0; degree of differentiation: medium and high differentiation = 1 and low differentiation = 0; vascular invasion: yes = 1 and no = 0; serum AFP level (ng/dL): ≥400 = 1 and <400 = 0; number of tumors: multiple = 1 and single = 0; maximum diameter of tumor (cm): ≥5 = 1 and <5 = 0; cirrhosis: yes = 1 and no = 0; nodule number: polynodule = 1 and single nodule = 0.

The article "Efficacy of TACE+Radiofrequency Ablation+Sorafenib in the Treatment of Patients with Recurrent Liver Cancer and Construction of Prediction Model" was retracted in 2023. Reasons: signs of a paper mill; compromised peer review; unreliable results or conclusions.

## Data Availability

The labeled dataset used to support the findings of this study is available from the corresponding author upon request.
